RETRACTED

# miR-18a-5p Targets FBP1 to Promote Proliferation, Migration, and Invasion of Liver Cancer Cells and Inhibit Cell Apoptosis

**DOI:** 10.1155/2021/3334065

**Published:** 2021-06-14

**Authors:** Shan Gao, Dongjie Zhu, Jian Zhu, Lianqiang Shen, Ming Zhu, Xuefeng Ren

**Affiliations:** Department of General Surgery, The First People's Hospital of Yuhang District, Hangzhou, Zhejiang 311100, China

## Abstract

Liver cancer is one of the most aggressive malignant tumors. It is significant to understand the molecular mechanism of liver cancer cells to develop new treatment plans. Studies have identified that FBP1 serves as a cancer inhibitor gene. To research the effect mechanism of FBP1 in liver cancer cells, bioinformatics analysis was performed to study its expression in liver cancer tissue. Survival analysis was also performed. Moreover, starBase database was applied to predict upstream regulatory genes of FBP1. Dual-luciferase assay was performed to testify their targeted relationship. The mRNA and protein expression levels of FBP1 in liver cancer cells were detected by qRT-PCR and western blot, respectively. Cell viability was analyzed by CCK-8 assay. The migratory and invasive abilities of cells were analyzed by Transwell assay. The apoptosis of liver cancer cells was detected by flow cytometry. The results showed that the expression of FBP1 was downregulated in liver cancer tissue and cells. FBP1 low expression was correlated with the poor prognosis of patients. miR-18a-5p could inhibit FBP1 expression. Overexpression of FBP1 could inhibit the progression of liver cancer cells and promote cell apoptosis. Overexpressing miR-18a-5p could promote the progression of liver cancer cells and inhibit cell apoptosis. However, overexpressing FBP1 simultaneously could reverse the effect. miR-18a-5p and FBP1 are expected to be candidates for liver cancer treatment.

## 1. Introduction

Liver cancer is a leading cancer worldwide with an increasing incidence rate. Despite progress in medicine, local treatment, and surgical treatment, it remains one of the most common causes for cancer-related deaths all over the world. Though more and more studies have been undertaken on liver cancer surgical treatment and molecular targeted treatment, the cure rate of this disease remains relatively low due to its high recurrent rate, high metastatic rate, and poor prognosis [1]. Therefore, it is pivotal to find a novel biomarker to predict liver cancer metastasis.

The gluconeogenic enzyme fructose-1, 6-bisphosphatase 1 (FBP1) is a key enzyme in gluconeogenesis, which can transfer FBP1 into fructose-6-phosphate [2]. More and more studies identified that FBP1 plays an important role in various cancers. For example, the methylation level of FBP1 promoter can be a new biomarker of the prognostic and therapeutic targets for patients with non-small-cell lung cancer [3]. Overexpressing FBP1 may inhibit the growth and migration of tumors via targeting HIF-1*α* in breast cancer cells [4]. FBP1 overexpression inhibits the proliferation and metastasis of cholangiocarcinoma cells via Wnt/*β*-catenin [5]. Loss of FBP1 promotes BET inhibitor resistance by undermining c-Myc expression in pancreatic ductal adenocarcinoma [6]. FBP1 is involved in epithelial mesenchymal transition (EMT), invasion, and metastasis of prostate cancer cells through regulating the MAPK signaling pathway [7]. Restoration of FBP1 suppresses EMT induced by Snail in liver cancer [8]. GSK343 induces programmed cell death via the suppression of FBP1 and EZH2 in osteosarcoma cells [9]. MAGE-TRIM28 complex targets FBP1 to promote the Warburg effect and liver cancer progression [10]. Loss of FBP1 promotes the invasiveness of liver cancer cells via the Warburg effect [11]. Inhibition of histone deacetylases restores FBP1 expression to suppress glucose metabolism and liver cancer growth [12]. Although there were imperfect studies about FBP1 in liver cancer [11], further exploration needs to be done about the mechanism of action of FBP1 in liver cancer cells.

miRNAs represented one of the most exciting fields in modern medicine because of their unique ability to regulate a huge complex network of gene expression [13, 14]. In recent years, there are an increasing number of studies about liver cancer and miRNAs. Li et al. [15] found that overexpressing miR-200c-5p inhibits the proliferation and metastasis of liver cancer cells, and it induces cell apoptosis and cell cycle arrest. Li et al. [16] found that miR-199b targets JAG1 to inhibit cell proliferation, migration, and invasion in liver cancer. Wang et al. [17] found that overexpressing miR-193a-5p can promote the proliferation of liver cancer cells and inhibit cell apoptosis. miRNA can also bind the 3′-untranslated region (UTR) of its target mRNA to mRNA expression [18]. miR-18a-5p can target SREBP1 to form a corepressor complex with Snail and HDAC1/2 to modulate EMT in breast cancer [19]. Besides, lncRNA can regulate the proliferation and invasion of tumor cells by targeting miR-18a-5p. For example, lncRNA CASC2 inhibits hemangioma cell growth by regulating the miR-18a-5p/FBXL3 axis [20]. lncRNA FENDRR inhibits colorectal cancer invasiveness by regulating the miR-18a-5p/ING4 axis [21]. Hence, it is helpful to explore the upstream regulatory gene of FBP1 and their regulatory mechanism in liver cancer.

RETRACTED

In this study, the expression of FBP1 was firstly bioinformatically analyzed. The upstream regulatory gene of FBP1 was then predicted. A series of cellular experiments were applied to explore the effects of FBP1 and its upstream gene on the progression of liver cancer cells. We explored and further clarified the regulatory mechanism of FBP1 in liver cancer cells, which laid a theoretical basis to find novel therapeutic methods.

## 2. Materials and Methods

### 2.1. Bioinformatics Analysis

Mature miRNA (normal: 50, tumor: 375) and mRNA (normal: 50, tumor: 374) and clinical data of TCGA-LIHC were downloaded from TCGA (https://portal.gdc.cancer.gov/) database. The *t*-test was applied to identify the expression of FBP1 in the normal tissue and tumor tissue. The samples were divided into the high-expression and low-expression groups according to the median FBP1 expression. Then, the “survival” package was used to perform survival analysis. Meanwhile, the correlation between FBP1 and clinical features was analyzed by one-way analysis of variance (ANOVA). Differential analysis was conducted on miRNAs using the “EdgeR” package (∣logFC | >2.0, padj < 0.01). The upstream regulatory gene was predicted by miRDB (http://mirdb.org/), mirDIP (http://ophid.utoronto.ca/mirDIP/index.jsp#r), TargetScan (http://www.targetscan.org/vert_72/), and starBase (http://starbase.sysu.edu.cn/) databases. The predicted miRNAs were intersected with upregulated differentially expressed miRNAs (DEmiRNAs). Pearson correlation analysis was carried out on the obtained miRNAs and FBP1, while the expression of miRNA was further clarified with *t*-test. At the same time, the above method was taken on target miRNA to perform the survival analysis.

### 2.2. Cell Culture

Human normal liver cell line L02 (MZ-0625) and liver cancer cell lines Hep3B (MZ-2124), HepG2 (ATCC HB-8065), SMMC7721 (MZ-0624), and MHCC97H (MZ-0692) were purchased from Ningbo Mingzhou Biotechnology Co., Ltd. All cells were cultured in Dulbecco Modified Eagle Medium (DMEM) supplemented with 10% fetal bovine serum (FBS) and then were maintained in an incubator under standard condition of 37°C and 5% CO_2_.

### 2.3. Cell Transfection

Synthesized miR-18a-5p-mimic, negative control (miR-NC), pWPXL-FBP1 (oe-FBP1), and blank plasmid pWPXL were purchased from GenePharma (Shanghai, China). According to the manufacturer's instruction, miR-18a-5p-mimic, miR-NC, and plasmid were transfected into HepG2 cell line using the Lipofectamine 2000 reagent (Invitrogen, Carlsbad, CA). Transfected cells were maintained with 5% CO_2_ at 37°C. After 24-48 h, cells were used for the following experiments.

### 2.4. qRT-PCR

Total RNA was extracted from the cell lines by TRIzol reagent (Life Technologies, Grand Island, NY, USA). To obtain cDNA templates, 1 *μ*g total RNA in each sample was applied for reverse transcription using miScript reverse transcription kit (Qiagen, USA) (37°C for 60 min; 95°C for 5 min). miRNA was reversely transcribed to cDNAs with miScript II RT kit (Qiagen, USA). mRNA was reversely transcribed as cDNA with PrimeScript RT Master Mix (Takara, Dalian, China). The expression of miRNA was detected with miScript SYBR Green PCR Kit (Qiagen, Germany). The expression of mRNA was detected with SYBR® Premix Ex Taq™ II (Takara Bio Inc., Shiga, Japan). The mRNA expression levels of miR-18a-5p and FBP1 were detected by qRT-PCR on the Applied Biosystems® 7500 Real-Time PCR Systems (Thermo Fisher Scientific, Waltham, MA). FBP1 and miR-18a-5p took *β*-actin and U6 as the internal references, respectively. Differences in expression level were compared with 2^-*ΔΔ*Ct^. Premier sequences are shown in Table 1.

RETRACTED

### 2.5. Western Blot Assay

Cells were lysed with RIPA lysis buffer (Beyotime, China) to obtain protein samples. Bicinchoninic acid (BCA) protein detection kit was used to measure the concentration of total proteins. Then, proteins were separated with 10% sodium dodecyl sulfate-polyacrylamide gel electrophoresis (SDS-PAGE) and then transferred onto a polyvinylidene fluoride (PVDF) membrane. Thereafter, the membrane was blocked with 5% blocking agent at room temperature for 1 h and washed with PBS 3 times. Then, the membrane was incubated with rabbit anti-FBP1 (1 : 2000, ab109732, Abcam, China) and rabbit anti-*β*-actin (1 : 1000, ab8227, Abcam, China) at 4°C overnight. Afterwards, secondary antibody goat anti-rabbit IgG H&L (HRP) (ab6721, Abcam, China) was incubated with the membrane at room temperature for 2 h after the membrane was washed 3 times. At last, the enhanced chemiluminescence (ECL) kit (GE Healthcare, Chicago, IL, USA) was applied for developing, with *β*-actin as an internal reference. The expression of protein was measured by Image Lab software (Bio-Rad Laboratories, CA, USA).

### 2.6. CCK-8

To evaluate cell viability, transfected cells were inoculated into 96-well plates at 1 × 10^5^ cells per well. After cells were inoculated for 1, 2, 3, and 4 d, cell proliferation was measured with CCK-8 detection (Dojindo, Japan). The absorbance of cells was determined at 450 nm.

### 2.7. Cell Migration and Invasion Assays

For invasion assay, Matrigel (BD Biosciences, San Jose, CA, USA) was added to the upper chamber to fabricate 24-well Transwell. Transfected HepG2 cells were seeded at 4 × 10^4^ cells/well and then cultured by serum-free medium. The lower chamber was added with medium with 10% FBS. After 24 h of incubation, noninvading cells were removed. Invading cells were fixed with 4% methyl alcohol for 0.5 h and stained with 0.1% crystal violet for 15 min. A microscope (Axioskop 40, Carl Zeiss AG, Dresden, Germany) was used to capture images in 5 random fields to calculate the numbers of invading cells. The upper chamber should not be added with Matrigel in Transwell migration assay, and the other procedures were the same with invasion assay.

RETRACTED

### 2.8. Cell Apoptosis Detection

Cell apoptosis was evaluated and analyzed by annexin V-FITC cell apoptosis detection kit and FACSCalibur flow cytometry (Becton Dickinson, CA, USA). Cells were washed with PBS 2 times, resuspended in binding buffer, and treated with annexin V-FITC for 15 min. Afterwards, propidium iodide (PI) was added. Stained cells were estimated by FACSCalibur (BD, USA).

### 2.9. Dual-Luciferase Assay

Luciferase reporter gene detection was performed on the above cell lines. Dual-luciferase reporter plasmids psiCHECK-FBP1 (Sangon Co., LTD., Shanghai, China) with 3′-UTR wild type (wt-FBP1) and 3′-UTR mutant type (mut-FBP1) of FBP1 were firstly constructed. Following the instruction of Lipofectamine 2000 (Invitrogen, USA) kit, miR-18a-5p-mimic/NC-mimic and psiCHECK-FBP1 wt/mut were cotransfected into HepG2 cells. Luciferase activity was measured by the Dual-Luciferase Reporter Assay System (Promega, USA) after cells were inoculated to 96-well plates for 24 h.

### 2.10. Statistical Analysis

All data were analyzed with GraphPad Prism 6.0 (La Jolla, CA), and each experiment was repeated 3 times (three technical repetitions and three biological repetitions). The results were represented as mean ± standard deviation (SD), and the comparison between the two groups was performed by *t*-test. Comparison of differences among multiple groups was done by analysis of variance (ANOVA). *p* < 0.05 represented a significant statistical difference.

## 3. Results

### 3.1. FBP1 Expression Is Significantly Downregulated in Liver Cancer Cells

Several studies indicated that FBP1 high expression inhibits the proliferation of liver cancer cells. To study the possible function of FBP1 in human liver cancer cells, FBP1 was chosen for research in this study. We firstly analyzed the TCGA-LIHC dataset and explored the expression and regulated molecular mechanism of FBP1 in liver cancer cells. According to TCGA-LIHC, FBP1 was significantly downregulated in liver cancer tissue (Figure 1(a)). Its low expression was positively correlated with poor prognosis (Figure 1(b)). Meanwhile, FBP1 was markedly correlated with the clinical stage and T stage (Figure 1(c)). The expressions of FBP1 in liver cancer cell lines (MHCC97H, HepG2, SMMC7721, and Hep3B) and human normal liver cell line (L02) were detected by qRT-PCR and western blot assays. It was found that the expression levels of FBP1 mRNA and protein were significantly downregulated in the liver cancer cell lines, wherein the expression in HepG2 cells was the lowest (Figure 1(d)). The above results represented that FBP1 was remarkably downregulated in liver cancer cells, and its low expression could affect the prognosis of patients. These results indicated that FBP1 may be involved in liver cancer progression. To better explore the effect mechanism of FBP1 in liver cancer cells, the HepG2 cell line with the lowest FBP1 expression was chosen for the following experiments.

RETRACTED

### 3.2. Overexpressing FBP1 Can Inhibit the Proliferation, Migration, and Invasion of Liver Cancer Cells and Promote Cell Apoptosis

To study the effect of FBP1 on the proliferation, migration, and invasion of liver cancer cells, we overexpressed FBP1 in the HepG2 cell line. The HepG2 cell line was transfected with oe-NC and oe-FBP1, respectively. Transfection efficiency of FBP1 in liver cancer cell line was detected by qPCR. It was shown that the expression of FBP1 in the oe-FBP1 group (compared with the oe-NC group) was significantly upregulated (Figure 2(a)). Thus, the cell line could be used in the following experiments. CCK-8 assay demonstrated that overexpressing FBP1 could inhibit the proliferative ability of liver cancer cells (Figure 2(b)). As indicated in Transwell assays, the migratory and invasive abilities of liver cancer cells were markedly reduced after overexpressing FBP1 (Figures 2(c) and 2(d)). Cell apoptosis assay showed that overexpressing FBP1 could promote the apoptosis of cancer cells (Figure 2(e)). The above results represented that overexpressing FBP1 could inhibit the proliferation, migration, and invasion of liver cancer cells and promote cell apoptosis. All data represented that FBP1 may be involved in the liver cancer cell progression.

### 3.3. miR-18a-5p Is Highly Expressed in Liver Cancer Cells and Significantly Negatively Correlated with FBP1

The above experimental results identified that FBP1 expression was downregulated in liver cancer. To testify the upstream regulatory mechanism of FBP1 in liver cancer, the differential analysis was performed using EdgeR. Next, 126 DEmiRNAs were obtained (122 upregulated miRNAs and 4 downregulated miRNAs) (Figure 3(a)). The upregulated DEmiRNAs were intersected with target genes predicted by miRDB, mirDIP, TargetScan, and starBase databases, and finally, miR-18a-5p was obtained (Figure 3(b)). The Pearson correlation between FBP1 and miR-18a-5p is shown in Figure 3(c). Significant negative correlation was found between them. The *t*-test indicated that miR-18a-5p was significantly upregulated in liver cancer tissue (Figure 3(d)). Survival analysis illustrated that miR-18a-5p high expression predicted poor prognosis of patients (Figure 3(e)). Afterwards, qRT-PCR was performed to detect the expression of miR-18a-5p in normal cell line and liver cancer cell lines. The result disclosed that miR-18a-5p expression was remarkably high in liver cancer cell lines (Figure 3(f)). All the above results indicated that FBP1 was markedly negatively correlated with miR-18a-5p. miR-18a-5p expression was significantly high in liver cancer cells, which was positively correlated with the poor prognosis of patients.

RETRACTED

### 3.4. miR-18a-5p Inhibits FBP1 Expression in Liver Cancer Cells

The above results indicated that miR-18a-5p was overexpressed in liver cancer cells and remarkably negatively correlated with FBP1. Later, we testified the targeted relationship between miR-18a-5p and FBP1. The binding sequence of FBP1 on miR-18a-5p was predicted with the starBase database (Figure 4(a)). It was testified by dual-luciferase assay that overexpressing miR-18a-5p could inhibit the luciferase activity of FBP1-wt, while no effect was discovered on the luciferase activity of FBP1-mut. It was identified that miR-18a-5p could target FBP1 (Figure 4(b)), and overexpressing miR-18a-5p could downregulate the expression of mRNA and protein of FBP1 in liver cancer cells (Figures 4(c) and 4(d)). The above experimental results verified that miR-18a-5p could target FBP1 and inhibit its expression in liver cancer cells.

### 3.5. miR-18a-5p Downregulates FBP1 to Promote the Proliferation, Migration, and Invasion of Liver Cancer Cells and Inhibit Cell Apoptosis

To identify the regulatory mechanism of miR-18a-5p and FBP1 in liver cancer cells, we constructed the overexpressed miR-18a-5p (miR-mimic) group and the simultaneously overexpressed FBP1 and miR-18a-5p (miR-mimic+oe-FBP1) group. The expression of FBP1 in liver cancer cells HeqG2 was detected by qPCR and western blot assays. The result indicated that FBP1 in the miR-mimic group was significantly declined, while no markedly changes were found in FBP1 expression after simultaneously overexpressing FBP1 and miR-18a-5p (Figure 5(a)). CCK-8 revealed that the proliferative ability of liver cancer cells was strengthened after overexpressing miR-18a-5p. However, the promoting effect of overexpressing miR-18a-5p on the proliferative ability of liver cancer cells was reduced after simultaneously overexpressing FBP1 and miR-18a-5p (Figure 5(b)). Transwell assay indicated that the migratory and invasive abilities of liver cancer cells were elevated after overexpressing miR-18a-5p. However, the promoting effect of overexpressing miR-18a-5p on the migratory and invasive abilities of cells was inhibited after simultaneously overexpressing FBP1 and miR-18a-5p (Figures 5(c) and 5(d)). Cell apoptosis was detected by flow cytometry. It was found that overexpressing miR-18a-5p could remarkably inhibit the apoptosis of liver cancer cells, while simultaneously overexpressing miR-18a-5p and FBP1 could inhibit the inhibitory effect of miR-18a-5p on cell apoptosis (Figure 5(e)). The above experimental results represented that miR-18a-5p could inhibit FBP1 expression to promote the proliferation, migration, and invasion of liver cancer cells and inhibit cell apoptosis.

RETRACTED

## 4. Discussion

Cancer is an extremely diversified and complex disease, which resulted from multiple genetic and epigenetic changes. For example, the expression levels of some mRNAs are closely related to cancer progression stages [22]. Liu et al. [23] found that the upregulation of RUNX1 inhibits the proliferation and migration of liver cancer via inhibiting VEGFA expression. Zhang et al. [24] found that overexpressing HIPK2 can inhibit the metastasis of esophageal squamous cancer cells. SOX4 inhibits WNT5a to regulate the invasion of bladder cancer cells [25]. Abundant references represented that FBP1 high expression inhibits the proliferation of liver cancer cells [7, 8, 12]. FBP1 promotes the development of ovarian cancer by promoting cell cycle transition and metastasis, and the expression of FBP1 increases with the development of ovarian cancer. Moreover, FBP1 cannot affect the apoptosis of ovarian cancer, but can strengthen cell cycle transformation. Therefore, FBP1 may promote the development of ovarian cancer by promoting cell cycle metastasis [26]. Thus, FBP1 was chosen for research. Mature miRNA and mRNA expression data as well as correspondent clinical data were downloaded from TCGA-LIHC in TCGA database. It was found that FBP1 was lowly expressed in liver cancer tissue and its low expression was relevant to the poor prognosis of patients. Meanwhile, FBP1 was significantly correlated with the clinical stage and T stage. A series of cytology assays testified that overexpressing FBP1 could inhibit the proliferation, migration, and invasion of liver cancer cells and promote cell apoptosis, which indicated that FBP1 was a cancer inhibitor in liver cancer.

Afterwards, the upstream regulatory miRNAs of FBP1 were obtained by bioinformatics analysis. Dual-luciferase assay also identified the binding relationship between them. More and more studies pointed out that miRNAs had a significant effect on the pathological mechanism and progression of human cancers. In this study, we firstly testified that miR-18a-5p could downregulate FBP1 in liver cancer cells, and highly expressed miR-18a-5p was relevant to the poor prognosis of patients. Many studies indicated that miR-18a-5p plays an important role in various cancers. For example, miR-18a-5p promotes the invasion and migration of osteosarcoma cells via directly targeting IRF2 [27]. The upregulation of miR-18a-5p has a positive effect on the proliferation and metastasis of renal tubular epithelial cancer cells and inhibits cell apoptosis [28]. lncRNA GASS regulates the proliferation, migration, and invasion of glioma cells by negatively regulating miR-18a-5p [29]. Upregulating lncRNA CASC2 may regulate miR-18a-5p/RUNX1 to inhibit the development of malignant melanoma [30]. The above studies show that miR-18a-5p plays a cancer promoter or cancer inhibitor role in various cancers.

RETRACTED

To verify the regulatory mechanism of the miR-18a-5p/FBP1 axis in liver cancer cells, we also established the simultaneously overexpressed miR-18a-5p and FBP1 (miR-mimic+oe-FBP1) group. Compared with the miR-mimic+oe-NC group, it was uncovered that overexpressing FBP1 could reverse the promoting effect of overexpressing miR-18a-5p on the malignant progression of the liver cancer cells. Zhang et al. [31] discovered that overexpressing miR-517a promotes the proliferation of liver cancer cells, while recovering FBP1 expression can inhibit the growth of cancer cells. The results of this study were similar to those of the study performed by Zhang et al., which disclosed that FBP1 could reverse the promoting effect of upstream regulatory genes on liver cancer cell growth.

Our study firstly discovered the molecular mechanism of the miR-18a-5p/FBP1 axis regulating liver cancer malignant progression. miR-18a-5p was upregulated in liver cancer cell lines and promoted liver cancer migration and invasion by inhibiting FBP1 expression. Ultimately, miR-18a-5p may be a potential drug therapeutic target and prognostic biomarker of liver cancer. But the downstream mechanism of FBP1 in liver cancer cells remains unclear, and specific mechanism of FBP1 in regulating tumor cell migration and invasion is unknown. Moreover, this study only designed cell functional experiments to verify the conclusion. Hence, we will continue to deeply investigate the detailed mechanism of FBP1 in regulating tumor cell migration and invasion in the following work. Besides, we will collect clinical tissue samples to construct a mouse model to further verify our hypothesis.

## Figures and Tables

**Figure 1:** FBP1 is significantly low in liver cancer cells. (a) Boxplot of the expression of FBP1 in the normal tissue and the tumor tissue samples, with green representing the normal group and red representing the tumor group. (b) Survival curve of FBP1, with abscissa representing the time (unit: year), ordinate representing the survival rate, green curve representing high expression, and red curve representing low expression. (c) Correlation between FBP1 and clinical features. (d) The expression of FBP1 in human normal liver cell line (L02) and 4 human liver cancer cell lines (MHCC97H, HepG2, SMMC7721, and Hep3B); ∗ represents *p* < 0.05 and ∗∗∗∗ represents *p* < 0.0001.

RETRACTED

**Figure 2:** Overexpressing FBP1 can inhibit the progression of liver cancer cells and promote cell apoptosis. (a) The transfecting efficiency of FBP1 in liver cancer cell HepG2 detected by qRT-PCR. (b) The proliferative ability of cells in different transfection groups (oe-NC and oe-FBP1) in liver cancer cell HepG2 detected by CCK-8. (c) The invasive ability of cells in different transfection groups (oe-NC and oe-FBP1) in liver cancer cell HepG2 detected by Transwell assay (×100). (d) The migratory ability of cells in different transfection groups (oe-NC and oe-FBP1) in liver cancer cell HepG2 detected by Transwell assay (×100). (e) The apoptotic rate of cells in different transfection groups (oe-NC and oe-FBP1) in liver cancer cell HepG2 detected by flow cytometry; ∗ represents *p* < 0.05.

**Figure 3:** miR-18a-5p is lowly expressed in liver cancer cells and negatively correlated with FBP1. (a) Volcano plot of DEmiRNAs in the normal group and the tumor group in liver cancer dataset in TCGA database, with red representing upregulated miRNAs and green representing downregulated miRNAs. (b) Venn diagram of predicted upstream miRNAs of FBP1 and DEmiRNAs. (c) Results of Pearson correlation analysis between FBP1 and its predicted upstream miRNAs (each dot represents a tumor sample). (d) Boxplot of the expression of miR-18a-5p, with green representing the normal group and red representing the tumor group. (e) Survival curve of the expression of miR-18a-5p on patient's prognosis, with the green line representing the high-expression group and the red line representing the low-expression group. (f) The expression of miR-18a-5p in human normal liver cell line (L02) and human liver cancer cell lines (MHCC97H, HepG2, SMMC7721, and Hep3B) detected by qRT-PCR; ∗ represents *p* < 0.05 and ∗∗∗∗ represents *p* < 0.0001.

**Figure 4:** miR-18a-5p can target and inhibit FBP1 expression in liver cancer cells. (a) Schematic diagram of binding sequence between miR-18a-5p and FBP1-wt and FBP1-mut. (b) Luciferase activity of FBP1 in liver cancer cell line HepG2 in different treatment groups detected by dual-luciferase assay. (c) The expression of FBP1 mRNA in liver cancer cell line HepG2 detected by qRT-PCR. (d) The expression of FBP1 protein in liver cancer cell line HepG2 detected by western blot; ∗ represents *p* < 0.05.

RETRACTED

**Figure 5:** miR-18a-5p targets and downregulates FBP1 to promote the proliferation, migration, and invasion of liver cancer cells and inhibit cell apoptosis. (a) The expression of FBP1 mRNA and protein in transfected liver cancer cells HepG2 (miR-NC+oe-NC, miR-mimic+oe-NC, and miR-mimic+oe-FBP1). (b) The proliferative ability of HepG2 cells in different treatment groups detected by CCK-8. (c) The invasive ability of HepG2 cells in different treatment groups detected by Transwell assay (×100). (d) The migratory ability of HepG2 cells in different treatment groups detected by Transwell assay (×100). (e) The apoptosis of HepG2 cells in different treatment groups detected by flow cytometry; ∗ represents *p* < 0.05.

**Table 1:** qRT-PCR primer sequences.

Gene	Premier sequence (5′ → 3′)
miR-18a-5p	F: 5′-ACACTCCAGCTGGGTAAGGTGCATCTAGTGC-3′
	R: 5′-CTCAACTGGTGTCGTGGAGTCGGCAATTCAGTTGAGCTATCTGC-3′
U6	F: 5′-CTCGCTTCGGCAGCACA-3′
	R: 5′-AACGCTTCACGAATTTGCGT-3′
FBP1	F: 5′-ACATCGATTGCCTTGTGTCC-3′
	R: 5′-CATGAAGCAGTTGACCCCAC-3′
*β*-Actin	F: 5′-TTGTTACAGGAAGTCCCTTGCC-3′
	R: 5′-ATGCTATCACCTCCCCTGTGTG-3′

## Data Availability

The data and materials in the current study are available from the corresponding author on reasonable request.
